# Plasma D-Dimer Levels Are Associated with Stroke Subtypes and Infarction Volume in Patients with Acute Ischemic Stroke

This article has been retracted.

**DOI:** 10.1371/journal.pone.0086465

**Published:** 2014-01-20

**Authors:** Wen-Jie Zi, Jie Shuai

**Affiliations:** 1 Department of Neurology, Xin Qiao Hospital, Third Military Medical University, Chongqing, P. R. China; St Michael’s Hospital, University of Toronto, Canada

## Abstract

**Background:**

It has been suggested that modestly elevated circulating D-dimer values may be associated with acute ischemic stroke (AIS). Thus, the purpose of this study was to investigate the association between plasma D -dimer level at admission and AIS in Chinese population.

**Methods:**

In a prospective observational study, plasma D-dimer levels were measured using a particle-enhanced, immunoturbidimetric assay on admission in 240 Chinese patients with AIS. The National Institutes of Health Stroke Scale (NIHSS) score was assessed on admission blinded to D-dimer levels.

**Results:**

Plasma median D-dimer levels were significantly (P = 0.000) higher in AIS patients as compared to healthy controls (0.88; interquartiler range [IQR], 0.28–2.11 mg/L and 0.31; IQR, 0.17–0.74 mg/L). D-dimer levels increased with increasing severity of stroke as defined by the NIHSS score(r = 0.179, p = 0.005) and infarct volume(r = 0.425, p = 0.000). Those positive trends still existed even after correcting for possible confounding factors (P = 0.012, 0.000; respectively). Based on the Receiver operating characteristic (ROC) curve, the optimal cut-off value of plasma D-dimer levels as an indicator for diagnosis of cardioembolic strokes was projected to be 0.91 mg/L, which yielded a sensitivity of 83.7% and a specificity of 81.5%, the area under the curve was 0.862(95% confidence interval [CI], 0.811–0.912).

**Conclusion:**

We had shown that plasma D-dimer levels increased with increasing severity of stroke as defined by the NIHSS score and infarct volume. These associations were independent other possible variables. In addition, cardioembolic strokes can be distinguished from other stroke etiologies by measuring plasma D-dimer levels very early (0–48hours from stroke symptom onset).

## Introduction

Acute ischemic stroke (AIS) is one of the major causes of death worldwide [1]. Timely intervention can dramatically improve outcome and reduce disability. It causes a great financial burden, since one-third of surviving stroke patients remain dependent in daily activities. Similarly, stroke places a tremendous burden on health resources in China [2].

D-dimer, the final product of plasma in-mediated degradation of fibrin-rich thrombi, has emerged as a simple blood test that can be used in diagnostic algorithms for the exclusion of venous thromboembolism. D-dimer levels have certain advantages over other measures of thrombin generation, because it is resistant to ex vivo activation, relatively stable, and has a long half-life [3]. The concentration of D-dimer reflects the extent of fibrin turnover in the circulation, because this antigen is present in several degradation products from the cleavage of cross linked fibrin by plasmin[4].

It has been suggested that modestly elevated circulating D-dimer values reflect minor increases in blood coagulation, thrombin formation, and turnover of cross linked intravascular fibrin (which is partly intra-arterial in origin) and that these increases may be associated with coronary heart disease [5]. D-dimer is known to be positively associated with coronary heart disease incidence and its recurrence, which is largely in dependent of conventional risk factors [5]–[6]. In addition, elevated D-dimer concentrations have been reported to be associated with cerebral venous sinus thrombosis [7], acute pulmonary embolism [8], spontaneous intracerebral hemorrhage [9], long-term neurologic outcomes in Childhood-Onset Arterial Ischemic Stroke [10]. Previous studies also have suggested that D-dimer levels may be associated specifically with subtypes [11], assessing prognosis [12]–[13] and unfavorable outcome in ischemic stroke patients. Some studies have suggested that D-dimer can be seen as an outcome predictor in ischemic stroke and an indicator of severity of traumatic brain injury [14]–[15].

Unfortunately, there has been little research on the associations between plasma D-dimer level and AIS in the Chinese patients. Thus, the purpose of this study was to investigate the association between plasma D-dimer levels at admission and subtypes, infarct size and severity in the Chinese patients with AIS.

## Methods

### Patients and Study Design

We conducted a prospective cohort study at the neurology department from December 2010 to October 2012. All patients with first-ever AIS were included. All patients were admitted within 24 hours of experiencing a new focal or global neurological event. Brain imaging (either CT or MRI) was performed routinely within 24 hours after admission. An AIS was defined according to the World Health Organization criteria [16]. We excluded patients with intracranial hemorrhage, malignancy, febrile disorders, acute or chronic inflammatory disease at study enrollment, coma or epileptic seizure activity, and patients who were anticoagulated before admission were also excluded. The onset time was defined as the time patients were last known to be without ischemic symptoms.

One hundred healthy people matched for age and gender were assigned to the healthy control group. Records of potential controls were reviewed by a neurologist (not an author) to exclude the presence of stroke, other types of diseases. This study was approved by the Institutional Review Board of The Xin Qiao Hospital, Third Military Medical University and informed written consent was obtained from each patient, family, or legal guardian.

### Clinical Variables

At baseline, demographic data (age and sex) and history of conventional vascular risk factors: hypertension, diabetes mellitus, dyslipidemia, other cardiac diseases (including acute myocardial infarction and angina), and cigarette smoking were obtained. Routine blood and biochemical tests, ECG, and a baseline brain CT/MRI scan were performed in all patients at admission. Stroke severity was assessed on admission using the National Institutes of Health Stroke Scale (NIHSS, the NIHSS score ranges from 0 to 34 and higher values reflect more severe neurological damage)[17] by a neurologist. Stroke subtype was classified according to TOAST (Trial of Org 10172 in Acute Stroke Treatment) criteria [18], which distinguished large-artery arteriosclerosis, small-artery occlusion, cardioembolism, other causative factor, and undetermined causative factor. The clinical stroke syndrome was determined by applying the criteria of the Oxfordshire Community Stroke Project: total anterior circulation syndrome (TACS); partial anterior circulation syndrome (PACS); lacunar syndrome (LACS); and posterior circulation syndrome (POCS) [19].

### Neuroimaging

MRI with diffusion-weighted imaging (DWI) was available in 183 stroke patients (76.3%). In those patients, DWI lesion volumes were determined by one experienced neurologist unaware of the clinical and laboratory results. The infarct volume was calculated by using the formula 0.5×a×b×c (where a is the maximal longitudinal diameter, b is the maximal transverse diameter perpendicular to a and c is the number of 10-mm slices containing infarct) [20]–[21].

### Blood Collection and Quantification

Blood samples of patients and controls were obtained at 7:00 AM in the next morning of the day of admission (within 0–6 [n = 131], 6–12 [n = 62], 12–24 [n = 26], and 24–48 [n = 21] hours from symptom onset). Patients’ blood samples were collected in the ward bedside in 5-ml vacuum tubes containing 0.5 ml buffered sodium citrate. Plasma aliquots were collected within one hour after randomization and centrifuged at 4000 g for 10 min at ambient room temperature. Plasma was then frozen at −70C until assayed.

D-dimer concentration was measured with a particle-enhanced, immunoturbidimetric assay in a calibrated SYSMEX7000 analyzer (Sysmex Corporation, Hyogo, Japan). The normal range of morning plasma D-dimer concentration in our hospital laboratory is 0–0.55 mg/L, which is slightly higher than other laboratory (0.25 mg/L [6]). The detection limit was 0.05 mg/L, and the dynamic range was from 0.07 to 35.2 mg/L. The intra-assay coefficient of variation [CV] and inter-assay CV were 1.5–3.4%, 2.6%–4.5%, respectively. Plasma levels of glucose, C-reactive protein (CRP), leucocyte count, prothrombin time (PT), activated partial thromboplastin time (APTT), thrombin time (TT) and fibrinogen (FBG) were also tested by standard method. For all measurements, levels that were not detectable were considered to have a value equal to the lower limit of detection of the assay.

### Statistical Analysis

Results are expressed as percentages for categorical variables and as medians (interquartile ranges, IQRs) for the continuous variables. Proportions were compared using the χ2 test, and the Mann–Whitney test or one-way analysis of variance (ANOVA) to compare continuous variables among groups. The relationship between serum D-dimer and others factors were determined using Spearman critical value rankings. Associations between NIHSS score and D-dimer were assessed using ordered logistic regression models in multivariate adjustment with possible confounders; ie, age, gender, stroke syndrome, stroke etiology, vascular risk factors and plasma levels of CRP, PT, APTT, TT and FBG. Associations between infarct volume and plasma D-dimer levels were also assessed using linear regression models in multivariate adjustment with the above confounders. Results were expressed as adjusted OR (odds ratios) with the corresponding 95% confidence interval (CI). Receiver operating characteristic (ROC) curves were utilized to evaluate the accuracy of D-dimer to predict AIS. Area under the curve (AUC) was calculated as measurements of the accuracy of the test. Two-sided P values of less than 0.05 were regarded as significant. All statistical analysis was performed with SPSS for Windows, version 18.0 (SPSS Inc., Chicago, IL, USA).

## Results

### Baseline Characteristics of Study Samples

During the inclusion period, 240 patients with AIS were included. The baseline characteristics of the 240 patients presenting with AIS are described in Table 1. Overall, in the study population, 166 (69.2%) were male and median age was 67 years (IQR, 53–76). The median NIHSS score on admission was 8 points (IQR, 5 to 11). The median time from symptom recognition to admission to hospital was 4.8 hours (IQR 2.2–10.1), and 199 patients (82.9%) were admitted within 12 hours of symptom recognition.

**Table 1:** Baseline characteristics of acute ischemic stroke patients and normal cases.

Characteristics	All(n = 240)	Normal cases (n = 100)	p^a^
Male sex (%)	166(69.2)	70(70.0)	NS
Age (years), median(IQR)	67(53–76)	66(52–77)	NS
Stroke severity, median NIHSS score (IQR)	8(5–11)	–	–
Infarct volume(mL, IQR; n = 183)	10(7–22)	–	–
Vascular risk factors no. (%)			
Diabetes mellitus	54(22.5)	–	–
Hypertension	172(71.7)		
Coronary heart disease	61(25.4)	–	–
Atrial fibrillation	55(22.9)		
Hypercholesterolemia	66(27.5)	–	–
Family history for stroke	52(21.7)	–	–
Smoking habit	49(20.4)	–	–
Clinical findings median(IQR)			
Temperature (°C)	37.0(36.4–37.4)	36.5(36.3–36.8)	<0.01
BMI (kg m^−2^)	24.8(23.2–27.4)	24.7(23.3–27.2)	NS
Heart rate (beats min^−1^)	82(72–91)	79(67–87)	NS
Systolic blood pressure(mmHg)	158(144–175)	127(112–134)	<0.001
Diastolic blood pressure(mmHg)	94(80–99)	80(75–86)	<0.01
Laboratory findings (median, IQR)			
Glucose(mmol L^−1^)	5.99(5.52–6.68)	5.45(4.76–5.93)	<0.001
C-reactive protein (mgL^−1^)	5.5(3.3–9.3)	3.2(2.5–6.6)	<0.01
Leucocyte count (×10^3^ m L^−1^)	8.2(6.3–9.4)	8.1(6.2–9.3)	NS
PT(second)	12.3(11.2–1.3.1)	11.1(10.6–11.6)	<0.01
APTT(second)	28.3(25.9–30.2)	26.9(24.5–28.6)	<0.01
TT(second)	18.3(17.7–19.1)	18.1(17.6–18.9)	NS
FBG(g L^−1^)	3.54(3.05–3.99)	2.93(2.34–3.66)	<0.01
D-dimer(mg L^−1^)	0.88(0.28–2.11)	0.31(0.17–0.74)	<0.001
Stroke syndrome no. (%)			
TACS	31(12.9)	–	–
PACS	95(39.6)	–	–
LACS	55(22.9)		
POCS	59(24.6)	–	–
Stroke etiology no. (%)			
Small-vessel occlusive	47(19.6)	–	–
Large-vessel occlusive	49(20.4)		
Cardioembolic	98(40.8)	–	–
Other	22(9.2)	–	–
Unknown	24(10.0)	–	–

IQR, interquartile range; TACS, total anterior circulation syndrome; LACS, lacunar syndrome; PACS, partial anterior circulation syndrome; POCS, posterior circulation syndrome; NIHSS, National Institutes of Health Stroke Scale; CRP, C-reactive protein; PT, prothrombin time; APTT, activated partial thromboplastin time; TT, thrombin time; FBG, fibrinogen.

^a^ *p* value was assessed using Mann-Whitney *U* test or χ2 test.

### Plasma D-dimer Levels and Stroke Characteristics

The results indicated that the Plasma D-dimer levels were significantly (P = 0.000) higher in AIS as compared to healthy controls (0.88; IQR, 0.28–2.11 mg/L and 0.31; IQR, 0.17–0.74 mg/L, respectively; Figure 1.). There were modest correlation that linked the plasma D-dimer levels to age(r = 0.212, p = 0.000), sex (r = 0.352, p = 0.000). PT and APTT were also correlated with the Plasma D-dimer levels (r = 0.211 and r = 0.205; P = 0.000, respectively).

**Figure 1:** Plasma D-dimer levels in acute ischemic stroke patients and control group. Mann–Whitney U-test. All data are medians and interquartile ranges (IQR). Significantly higher in stroke patients as compared to those in normal cases (p = 0.000).

Plasma D-dimer levels increased with increasing severity of stroke as defined by the NIHSS score. There were positive correlation that linked the levels of D-dimer to the NIHSS (r  = 0.179, p = 0.005; Figure 2a.), FBG (r  = 0.346, p = 0.000; Figure 2b.) and CRP levels (r  = 0.261, P = 0.000; Figure 2c.). There was still a significant positive trend between plasma D-dimer levels and NIHSS score (P = 0.012), using ordered logistic regression after multivariate adjustment for possible confounders: age, gender, time to admission, stroke syndrome, stroke etiology, vascular risk factors and plasma levels of CRP, PT, APTT, TT and FBG.

**Figure 2:** Correlation between plasma D-dimer levels and others predictors. (a) Correlation between plasma D-dimer levels and the National Institutes of Health Stroke Scale (NIHSS) score; (b) Correlation between the plasma D-dimer levels and fibrinogen levels; (c) Correlation between plasma D-dimer levels and CRP; (d) Correlation between plasma D-dimer levels and infract volume.

In patients for whom MRI data were available (n  = 183), there was a positive correlation between levels of D-dimer and the infarct volume (r  = 0.425, P = 0.000; Figure 2d.). There was still persists a significant positive trend between plasma D-dimer levels and infarct volume (P = 0.000), after adjustment for the same above covariates. In addition, D-dimer levels were significantly lower in patients with LACS 0.55 mg/L (IQR 0.21–1.56 mg/L) compared with patients with PACS 0.92 mg/L (IQR 0.32–2.06, p<0.001), POCS 0.88 mg/L (IQR 0.29–2.16, p<0.001) or TACS 0.90 mg/L (IQR 0.28–2.08, P<0.01).

### Plasma D-dimer Levels and Stroke Etiology

Significant *stroke etiology* differences in plasma D-dimer levels were observed ((analysis of variance [ANOVA]: p = 0.000); See the Figure. 3). D-dimer levels in patients with cardioembolic stroke (2.17 mg/L (IQR, 1.24–3.48)) were significantly higher as compared with small-vessel occlusive stroke (0.59 mg/L (IQR, 0.25–0.96)), large-vessel occlusive stroke (0.56 mg/L (IQR, 0.22–0.95)), other stroke (0.25 mg/L (IQR, 0.14–0.41)) and unknown stroke (0.29 mg/L (IQR, 0.18–0.68)); P = 0.000, respectively. A multiple regression model also demonstrated a significant correlation between stroke category and D-dimer levels (P* = *0.006).

**Figure 3:** Plasma D-dimer levels in different *etiology of* acute ischemic stroke patients. Significant differences in plasma D-dimer levels were observed (analysis of variance [ANOVA]: p = 0.000).

D-dimer (medians) were higher in patients with cardioembolic strokes than in those with other etiologies (2.17 vs. 0.47 mg/L, P = 0.000). Based on the ROC curve, the optimal cut-off value of plasma D-dimer levels as an indicator for diagnosis of cardioembolic strokes was projected to be 0.91 mg/L, which yielded a sensitivity of 83.7% and a specificity of 81.5%, the area under the curve was 0.862(95%CI, 0.811 – 0.912). See the figure 4. In this process, the positive predictive value was 83.9%, and the negative predictive value was 87.8%.

**Figure 4:** Receiver operating characteristic (ROC) curves were utilized to evaluate the accuracy of D-dimer levels to predict cardioembolic strokes.

## Discussions

In our study, we reported that plasma D -dimer levels were significantly increased in cases of first AIS compared to age and gender matched healthy controls. Our main findings were that D-dimer levels were in correlation with stroke subtypes and could be seen as an indicator for diagnosis of cardioembolic stroke. Furthermore, we found that the D-dimer levels increased with increasing severity of stroke as defined by the NIHSS score and infarct volume. Those positive trends still existed even after correcting for possible confounding factors.

Our findings were consistent with results of previous prospective studies showing that D-dimer levels were elevated in the acute phase of AIS compared with the healthy control population [22]–[23]. Smith et al [24] reported that D-dimer could predict incident stroke in the general population, even though no significant association was seen in the Three-City French cohort study [25]. In addition, a sex and age-related increase in D-dimer levels were noted between stroke patients and controls [26], which was in accordance with our work. In another study [27], elevated D-dimer was related to stroke severity on admission and poor outcome at discharge. We also found that D-dimer was related to stroke severity.

D-dimer levels have been shown to be associated with cardioembolic strokes [28]–[29], yet their significance in acute stroke remains to be determined. Overall, our data provided a detailed description of plasma D-dimer levels in correlation with stroke subtypes, and D-dimer levels were significantly higher in cardioembolic patients than in noncardioembolic AIS patients or healthy control subjects, which was in accordance with prior works [26]. Furthermore, Dougu et al [30] have also reported that D-dimer level of >1.6 mg/L may indicate a high possibility of cardioembolic. Takano et al [31] reported a D-dimer cut-off point of 300 ng/mL for distinguishing cardioembolic stroke from atherothrombotic infarction (ATI) and lacunar infarction (LI), yielding a sensitivity of 80% and a specificity of 77%. Another study proposed that the optimal D-dimer cut-off point for discriminating between the presence and absence of a cardioembolic source be 2.00 μg/mL to yield a specificity of 93%, a sensitivity of 59%, a positive predictive value of 73%, and a negative predictive value of 88% [32]. In our study, the optimal cut-off value of plasma D-dimer levels as an indicator for diagnosis of cardioembolic strokes was projected to be 0.91 mg/L, which yielded a sensitivity of 83.7%and a specificity of 81.5%, the area under the curve was 0.862(95%CI, 0.811 - 0.912). These reports appeared to suggest that assay of D-dimer levels in the acute stage of AIS can be useful in distinguishing cardioembolic strokes. Increased D-dimer level is hypothesized to be indicative of thrombus formation within the left Atrium and is the key factor of cardiac embolism onset [33].

This study showed that elevated levels of D-dimer in the 24-hour after AIS were associated with brain infarct volume independent of other clinical and laboratory variables. These results were in accordance with the results from other studies showing that D-dimer were associated with brain infarct [34], and had a statistical correlation to infarct volume [35]–[36].

There are several plausible mechanisms through which D-dimer levels could be closely related to stroke. Firstly, increased D-dimer levels may reflect ongoing thrombus formation within cerebral vessels or may be a marker of systemic hypercoagulability[37]. Furthermore, thrombi formed in hypercoagulable states such as high D-dimer levels may be resistant to the endogenous fibrinolytic system [38]. Secondly, some markers of hemostatic function are acute-phase reactants; D-dimer is one of these markers. There is, in fact, some evidence that fibrin degradation products, including D-dimer, may act to stimulate the inflammatory process [39], and this might provide a further pathological mechanism through which D-dimer is linked to progressing stroke [40]. There is some evidence that D-dimer itself stimulates monocyte synthesis and release of proinflammatory cytokines such as interleukin- 6[41]. Elevated systemic inflammation reflected by high D-dimer levels could also contribute to the stroke severity [42]. Activated inflammation and activated coagulation, in concert with each other, may contribute to the development of stroke. Thirdly, because D-dimer is one of the acute phase reactants, it is possible that elevated D-dimer levels in patients with stroke may be the result rather than the cause of stroke. Although D-dimer was significantly correlated with baseline infarct volume, D-dimer was associated with severity independently of infarct volume. Thus, we consider that it is less likely that elevated D-dimer is merely an epiphenomenon of development of stroke.

Some limitations of this observational study merit consideration. Firstly, without serial measurement of the circulating D-dimer levels, this study yielded no data regarding how long after the initiation of clot formation D-dimer levels become elevated or for how long they remain elevated in circulation. Secondly, follow-up data are lacking. Welsh et al [42] have reported that D -dimer were independently associated with poor outcome in acute ischemic stroke, and Barber et al [37] suggested that other potentially important factors were taken into consideration, fibrin D-dimer levels independently predicted progressing stroke. Further studies are needed to determine whether elevated D-dimer predicts outcomes after a stroke in our population. Thirdly, a number of different commercial D-dimer assays are available, and so our results may not necessarily be generalized to all assays. Furthermore, D-Dimer level is very rarely elevated in healthy individuals, however, may increase in many illnesses and physiological conditions associated with thrombosis and thrombolysis [43]. These patients may have had widespread vascular disease before stroke onset and are, therefore, likely to have increased pre-event levels when compared with population controls. We cannot exclude the possibility that plasma D -dimer increased under those state.

In conclusion, we have shown that plasma D-dimer levels increased with increasing severity of stroke as defined by the NIHSS score and infarct volume and these associations were independent of inflammation and other possible variables. In addition, cardioembolic strokes can be distinguished from other stroke etiologies by measuring plasma D-dimer levels very early (0–48hours from stroke symptom onset).
